This article has been retracted.

# Study on Health Care Service Standard of Chronic Disease Management Based on Process Reengineering and the Delphi Method

**DOI:** 10.1155/2022/6713140

**Published:** 2022-09-20

**Authors:** Jing Zhao

**Affiliations:** Nursing Department, West Anhui Health Vocational College, Lu'an 237000, China

## Abstract

The Delphi method is also called an expert consultation method, scientifically measuring the objectivity, practicality, and authority of the metric. This study aims to build a standard plan for chronic disease management care services in hospitals and guide the development of chronic disease management care services. This article proposes a chronic disease management nursing experiment, further revises the current hospital chronic disease management nursing service, redesigns the program, compiles the chronic disease management hospital nursing standard list according to the new program, and uses expert suggestions to modify the standard program items. It adopts a preliminary expert inquiry table, submits Delphi expert inquiry, and constructs a chronic patient prevention strategy for clinical nursing practice to learn from the reference for guiding the actual specific situation of nursing, providing evidence basis and practice guidance. More than 40 initial standards were listed, which were reduced to 30 after revision. The importance of the indicators to different experts was 3.56 to 4.85 points. The coordination coefficient is 0.180~0.356. Finally, after discussion by all parties, more than 40 specific indicators including the size of the new standard have been determined, which provides a great theoretical basis for the establishment of a new type of hospital chronic disease management and nursing service standard in my country. Based on process reconstruction and the Delphi method determined by the hospital chronic disease management nursing service standards, clear normative and operability can provide basis for the development of chronic disease management nursing services.

## 1. Introduction

Chronic disease does not specifically refer to a certain disease, but a description of symptoms that are hidden, take long time, complicated, and difficult to recover. It is a general term for diseases that have long-term harm to health but do not cause infection. If it is not treated for a long time, it is also will cause serious harm to the human body. Chronic diseases are likely to lead to organ failure, more likely to cause pulmonary fibrosis, asthma, and decreased lung function. Up to now, the number of people suffering from different types of chronic diseases in our country has exceeded 400 million, which has become a large part of our country's annual death toll. Chronic diseases may become very serious; safety and health problems, social problems, economic problems and so forth affect our country's development. To prevent chronic diseases, it is necessary to have reasonable diet, moderate exercise, quit smoking, limit alcohol, and have psychological balance. With the extensive application of the Delphi method in various fields, this method is also constantly developing and improving. It was not until the middle of this century that the Delphi method began to be used in medicine. Subsequently, the scope has gradually expanded in recent years. The Delphi method has become the most commonly used forecasting method. It is often used in the military industry to develop market demand population forecasting, field, medical and health forecasting research, project evaluation, and so forth. The Delphi method is widely used in medical treatment, prevention, health care, and other fields. The application of the Delphi method in the hospital's chronic disease management and nursing services in this study is also a very bold attempt to fit the background of the current era.

At present, various hospitals in our country are gradually opening up chronic disease management and nursing services, but because of the short development cycle of chronic disease management and nursing services, many processes are still in the exploratory stage, and the links and special requirements are not clear. This is in the hospital and obstacles to the development of chronic disease management in nursing services. To eliminate this obstacle, we must adhere to the guiding ideology of participation of the whole people, focus on prevention, combination of prevention and treatment, active initiation, and steady progress. This study uses the process reengineering method to update the traditional chronic disease management and nursing services. Process reengineering is also called business process reengineering, and it is often abbreviated as “BPR”. Many business processes have been redesigned and revised. The ultimate goal is to optimize and improve the quality of external products or services. New management methods and theories for reducing operating costs and improving the timelines of business processes were found in the 1890s. This study is based on the management of chronic diseases and the procedures of our hospital's nursing services. Brainstorming is used to redesign the hospital's chronic disease management system and nursing process. Then, expert advice is used to establish chronic diseases in the management of hospitals and nursing services. Chronic disease and nursing hospital service management standardization and improvement plan provides an objective basis for improving the management of chronic diseases and nursing services in hospitals in our country.

Process reengineering (PR) is a newly introduced process management method; it pays close attention to all processes related to achieving organizational goals. Although originally developed and applied for the private sector, PR is expected to become a convenient tool for the transformation of the public sector 263 organization (PSO) workflow, especially in this era of information and communication technology. Fatile Olufemi J conducted an X-ray examination of the PR of the African Public Sector Organization (APSO), highlighting lessons learned from the private sector. This article uses a descriptive method to verify and modify the existing theoretical models related to the interpretation of PR in APSO. Fatile Olufemi J observed that APSO is different from a private sector organization (PrSO). PSO has failed in adopting PR and performing logically related tasks in a way that achieves well-defined results. The private sector can use personal interests to motivate the members of the organization and stimulate the enthusiasm of the members of the organization to accomplish the established strategic goals. It further reveals that APSO's poor PR hinders Africa from achieving high performance, efficient service delivery, public satisfaction, efficient resource management, and sustainable development. The conclusion of this article is that if APSOs can reduce excessive bureaucracy, as advocated by contingency theory (CT), and learn more from the private sector in preparing for and adapting to environmental changes and transformations, they can completely adopt PR. The document recommends including the availability of information technology (IT) infrastructure and the willingness of government representatives to deploy new technologies through adequate support for information technology companies and prioritizing the high system requirements of IT applications. APSO managers should be given the power to implement changes when needed, without any form of influence. In addition, attention should be paid to the future of PSO. Citizens as its customers should be highly respected and not regarded as “people in need”. Finally, APSO should accept the fundamental changes associated with PR, especially by ensuring that promotions are based on performance and not just qualifications. However, he did not conduct research on the methods and experience of developed regions, then combined with the actual situation in Africa, and finally reached a conclusion [1]. Patients with rotator cuff lesions in the healthcare system do not always receive high-quality care. When patients receive care that is accessible, appropriate, acceptable, effective, efficient, and safe, high-quality care will appear. The purpose of the Eubank BH research is twofold: (1) Develop a clinical pathway algorithm that proposes a step-by-step process for making decisions for the pathological diagnosis and treatment of the rotator cuff in primary, secondary, and tertiary medical institutions. The development of treatment algorithms and decision tree methods provides a step-by-step sequence that can improve the quality, consistency, and coordination of care throughout the care continuum. (2) Establish clinical practice guidelines for pathological diagnosis and treatment of the rotator cuff to provide information for the decision-making process in the algorithm. Usage of the three steps improved the Delphi method to build consensus. Fourteen experts from sports therapy, physical therapy, sports medicine, and orthopedic surgery were invited to participate as expert groups. In the first round, 123 best practice statements were distributed to the group. Team members were asked to mark “agree” or “disagree” next to each statement and provide comments. His experiment only had a round of discussion, and the results obtained were too few to explain the public [2]. Economically disadvantaged individuals with chronic diseases have high rates of hospitalization (IP) readmission, and emergency department (ED) after their initial hospitalization. The purpose of this study is to explore the complexity of chronic diseases, health system integration (accommodation of responsible medical institutions [ACO] hospitals), availability of medical management interventions (membership of managed medical institutions [MCO]), and utilization of health care after 90 days of discharge. Hewner used unidentified Medicaid claims data from two counties in western New York. The study population consisted of 114,295 individuals who met the inclusion criteria, of which 7,179 had an index hospitalization in the first 9 months of 2013. According to the existence of 12 common diseases, individuals are assigned to three disease complex parts. The 30-day hospitalization (IP) readmission rate ranges from 6% in the nonchronic part to 12% in the complex part of chronic disease and 21% in the complex part of organ system failure. The hospitalization rate (inpatient and emergency department) of MCO and ACO patients is lower than that of patients charged for service. The complexity of chronic diseases, initial hospitalization at an institution belonging to the ACO, MCO membership, female, and longer hospital stays are related to the significantly longer readmission time in the first 90 days, that is, less readmission time. The results of Hewner S further prove that high-value post-discharge utilization (less IP or ED hospitalization and early outpatient follow-up) require population-based transitional care strategies to improve continuity between environments and take into account the medical assistance population disease complexity. Hewner S's research only stays at the theoretical level, without conducting specific experiments and obtaining results, which can finally support his theory [3].

This article deeply researches the establishment of chronic disease management and nursing service standards and uses the PR and the Delphi methods to update the current number of chronic patients and treatment and nursing methods in my country. We strictly followed the PR method and set up the first BPR team at the beginning of the experiment, composed of experienced experts from different departments. After brainstorming, it was redesigned, and a new process was created. The first three steps of scientific and reliable PR methods were well completed. This has laid a good foundation for the establishment of chronic hospital disease management service standards. The Delphi method is an essential expert research method, and the experts interviewed in this experiment have long-term theoretical and practical experience and have treated many patients with chronic diseases. They have a great say.

## 2. PR and the Delphi Method

### 2.1. Process Reengineering

Process reengineering (PR) is a new design process that was proposed by two famous American scientists, Michael Hammer and James Champy, and it reached its peak in 1990, as shown in Figure 1. A new governance process as an organizational activity to analyze was designed and the organizational process in a basic and thorough manner was planned [4]. Related organizational changes were managed to track performance and help the company grow significantly [5]. The focus of the new business design is to select multiple business processes that are critical to business activities and redesign them to improve operational efficiency [6]. It implements process management by sorting out and streamlining enterprise and industrial processes. The goal is to achieve significant improvements in cost, quality, outsourcing, and timeliness. The core of the redesign process is the business process that focuses on customer satisfaction. The main idea is to break the method of organizing management departments based on the company's operating conditions. In chronic disease nursing, follow-up nursing PR creates a chronic disease nursing service model with nursing professional characteristics and replaces it with a business process, plans new business management processes, and verifies the overall business process. Looking for the right person in the world is not the most suitable person. Competition and disputes between brands will gradually weaken, replaced by competition between the strength and efficiency of the company's value chain. The company needs to invest heavily, handle it carefully, protect, and continuously improve its assets.

Nowadays, all parties at home and abroad do not have an accurate definition of PR, and they have different models of it [7], but there are probably three models that are generally recognized and widely circulated: (1) Michael Hamer's four-stage model: the first stage, rebuild a new team; the second stage, establish a new goal; the third stage, design a new program; and the fourth stage, implement a new program [8]. (2) Joe and Roland's five-stage model: the first stage, build the environment; the second stage, analyze the original plan and ask questions; the third stage, rebuild the organizational structure; the fourth stage, the replacement stage; and the fifth stage, the realization goal [9]. (3) William J﹒Heidinger's six-stage model: the first stage, propose a new idea; the second stage, start the process; the third stage, analyze the original process; the fourth stage, design a new process; the fifth stage, rebuild a new process; and the sixth stage, evaluation and summary [10]. However, in our application, we are still using Michael's four-stage model. The specific conditions of the three models are shown in Figure 2.

The application of PR and the Delphi method to the research and application of chronic disease management and nursing technology can more fully and accurately use health data sets, making the effect of data mining more ideal [11]. The Delphi method makes the prediction opinions of the expert group tend to be concentrated and finally makes a prediction conclusion that is in line with the future development trend of things.

(1) $$\begin{array}{c} s_{t}=b*x_{t}+\left(1-b\right)*s_{t-1}, \end{array}$$

(2) $$\begin{array}{c} s=\sqrt[{x}]{f}*\frac{m}{b-1}{\left(b_{1}-b_{2}\right)}^{n}, \end{array}$$

Analysis has a smoothing effect on the actual sequence.

(3) $$\begin{array}{c} s_{t}=f\left(p*x_{t}+m*s_{t-1}\right). \end{array}$$

In the above formula, *f* is the input layer, *m* is the hidden layer, and *p* is the output layer. RNN leads to an exponential increase in the amount of calculation, which increases the time cost of the model. Therefore, the RNN model is not directly used for long-term memory calculations. On the basis of the original RNN network, LSTM adds valve nodes in each layer, which helps overcome the long-term memory problem that RNN is not good at and has been widely used [12].

(4) $$\begin{array}{c} f_{x}=\mathrm{sgn}\left(\overset{m}{\underset{a=1}{\sum }}x_{t}y_{t}\left(m_{a}*m\right)+b\right), \end{array}$$

(5) $$\begin{array}{c} f_{n}=\left(f_{1},f_{2},f_{3}\cdots \cdots f_{xy}\right)+a*b. \end{array}$$

Through the kernel function, the low-dimensional space can be converted into high-dimensional space and then classified by the abovementioned SVM classification model, where *x* and *y* represent data with different structures, *t* represents the growth rate, and *b* represents the prevention of lesions. Through conversion, the low-dimensional inseparable first is converted to the high-dimensional linearly separable [13].

(6) $$\begin{array}{c} a=\frac{1}{m}\overset{m}{\underset{i=1}{\sum }}\left(t_{u}^{i}-t_{v}^{i}\right). \end{array}$$

The matching criteria are given according to the above formula, using the PR and the Delphi method for chronic disease management and nursing services, and in-depth research on this service.

(7) $$\begin{array}{c} sim\left(c,m\right)={NNE}^{2}\left[E_{a},E_{b}\right]. \end{array}$$

One group represents the reconstruction methods in *C* and *m*. *a* and *b* are the tf-idef vector and the maximum average difference, respectively. The similarity between *c* and *m* can be freely defined. Through transfer learning, time-consuming and laborious processing costs can be greatly reduced. After a period of labeling and confirmation through transfer learning, a suitable training set can be established [14].

The relationship between the family burden and the number of patients can be expressed as follows:

(8) $$\begin{array}{c} ss=\frac{fa}{fa+pn}\underset{a}{\sum }b^{2}. \end{array}$$

### 2.2. Delphi Method

The Delphi method is an essential expert research method. The American RAND Corporation used this method for the first time in its forecast in 1964, soliciting anonymous expert opinions. After repeated information exchanges and revision suggestions, the opinions of the experts will gradually become consistent and finally start from the comprehensive perspective of the experts. The Delphi method is widely used in nursing, including clinical nursing, nursing education, nursing management, nursing research, community nursing, and so on. Quantitative and quantitative evaluations of object evaluation have been created [15]. The biggest advantage of this method is that it is simple and easy to use, without tedious mathematical modeling and can effectively predict the unknown or future state of the research object in the absence of sufficient statistical data. In addition, it has no similar historical facts to learn from. This is a leap in quality analysis, which goes beyond the field of pure qualitative or quantitative analysis. The Delphi method can synthesize the expert opinions of experts and expand the thinking of scientific and reasonable decision-making. With the wide application of laws in various fields, this method is constantly developing and improving. It was not until the middle of this century that the Delphi method began to be used in medicine and gradually expanded its scope. In the past few years, the Delphi method has become the most widely used forecasting method. It is often used for military machinery industry development, market demand, population forecasting, industry, medical and health forecasting, and evaluation of research projects in my country. The Delphi method is widely used in medical treatment, prevention, health care, and other fields [16] such as medical technology and education, primary health care technology design, technology evaluation, and technology and financial demonstration. The Delphi method is shown in Figure 3.

The Delphi method has the following characteristics:

1. Anonymity: The experts who participated in the prediction in the experiment did not know who participated in the prediction. They completed the prediction on their own and exchanged opinions anonymously. The Delphi method uses the form of anonymous surveys, which can overcome the shortcomings of the research method of meeting with experts and constitute risky meeting trends, atmosphere, and other psychological effects on the principles [17].
2. Feedback: The Delphi method uses an anonymous form. Therefore, experts will not communicate with each other, but rely on a round of research. Expert opinions are often scattered, making it difficult to draw conclusions. The invited experts understand the summary of each consultation cycle and the opinions of other experts. The organizer should classify, analyze, and collect the results of each round of consultation and make recommendations to each recipient in the next round of experts for further comments. Their opinions are based on the new questionnaire [18].
3. Statistical: When the Delphi method is used in the research, the evaluation or prediction of the research topic is not done by individual researchers or experts. However, a group of experts participated and was sent to many experts to perform statistical processing on the response. The results obtained using the Delphi method are statistical in nature and often appear in the form of probability. It not only reflects the strength of expert opinions but also clearly reflects the level of expert opinion [19]. The responses of many experts had to be statistically processed.

According to the rating of the indicators by experts, SPSS16.0 statistical software is used to record the consultation results, analyze the data, and calculate the average value of each indicator. The full score, frequency variation coefficient, the coordination coefficient of opinions, the enthusiasm of experts and participating experts, power, the degree of enthusiasm of the experts, and so forth are generally expressed by the recovery rate of the questionnaire. The more questionnaires are recovered, the higher the degree of enthusiasm of the experts. The weight percentage method is used to calculate and display the weight coefficient of each indicator in the system. Expert authority level (*C*_R_):

(9) $$\begin{array}{c} C_{\text{R}}=\frac{C_{\text{A}}+C_{\text{B}}}{2}. \end{array}$$

Among them, *C*_R_ represents the authority of the expert, *C*_A_ represents the basis for the expert to make a judgment, and *C*_B_ represents the expert's familiarity with the indicator. Normally, the larger *C*_R_ is, the higher the degree of expert authority [20].

Arithmetic average of the concentration of expert opinions:

(10) $$\begin{array}{c} M_{j}=\frac{1}{m}\overset{m_{j}}{\underset{i=1}{\sum }}C_{ij}. \end{array}$$

*M_j_* is the arithmetic average of all evaluations of the *j* (*j* = 1, 2, ⋯, *n*) program; *m_j_* is the number of experts participating in the evaluation of the *j* program; *C_ij_* is the *i*th (*i* = 1, 2, ⋯, *m*) scoring value of the *j*th scheme by the experts. The value of *M_j_* is 0–100 points. The larger the value of *M_j_*, the greater the relative importance of the program [21].

The full score frequency of a program refers to the ratio of the number of experts who give full marks to the program to the total number of experts who have evaluated the program. The calculation formula is as follows:

(11) $$\begin{array}{c} {K_{j}}^{\prime }={m_{j}}^{\prime }/m_{j}. \end{array}$$

*K*_*j*_′ is the frequency of full marks for plan *j*, and m_*j*_′ is the number of experts who give full marks to plan *j*; *m_j_* is the number of experts who participated in the evaluation of plan *j*; the value of *K*_*j*_′ is 0–1, and the larger *K*_*j*_′ is; the number of experts who give full marks to plan *j* the more relative, the greater the relative importance of the program [22].

The evaluation level sum of the program is the arithmetic sum of the evaluation levels of the experts to evaluate the program.

(12) $$\begin{array}{c} S_{\text{j}}=\overset{m_{j}}{\underset{i=1}{\sum }}R_{ij}. \end{array}$$

*S_j_* Is the evaluation level sum of the *j* scheme, and *R_ij_* is the evaluation level of the *i*th expert on the *j*th scheme. The smaller the value of *S_j_*, the greater the relative importance of the scheme [23].

The degree of coordination of expert opinions is usually expressed by the coefficient of variation and the coefficient of coordination. The calculation formula of the coefficient of variation is as follows:

(13) $$\begin{array}{c} V_{\text{j}}=\frac{\delta_{j}}{M_{j}}. \end{array}$$

*δ* is the standard deviation of the *j* index score, and *M_j_* is the arithmetic mean of the J index score.

The calculation formula of the coordination coefficient is as follows:

(14) $$\begin{array}{c} W=\frac{12}{{\text{m}}^{2}\left(n^{3}-n\right)-m\sum_{i=1}T_{i}}\overset{m}{\underset{j=1}{\sum }}d_{j}^{2}. \end{array}$$

*W* is the coordination coefficient, *n* is the number of indicators, *m* is the number of experts, *d_j_* is the difference between the index level and the arithmetic mean of the sum of all index levels, and *T_i_* is the correction coefficient.

Significance test formula of coordination coefficient is as follows:

(15) $$\begin{array}{c} {\text{x}}^{2}=\frac{1}{mn\left(n+1\right)-\left(1/n-1\right)\sum_{i=1}^{m}T_{i}}\overset{n}{\underset{j=1}{\sum }}d_{j}^{2}. \end{array}$$

### 2.3. Hospital Chronic Disease Management and Nursing Services

Chronic disease is a general term for diseases that have long-term harm to health but do not cause infection. It does not specifically refer to a certain disease, but a description of symptoms that are hidden, take a long time, are complicated, and are difficult to recover [24]. Although the chronic disease may not be as strong as the acute disease reaction, when the patient's chronic disease is not treated for a long time, it will also cause serious harm to the human body. Members of the public relations team use brainstorming to distinguish chronic disease management procedures and hospital services [25]. Public health service projects focus on primary medical and health service institutions, including health centers, community health service centers, and so forth The results of domestic and foreign literature review and the Web browsing platform are combined. The establishment of chronic disease nursing management institutions, chronic disease patient registration institutions, and establish personal chronic disease files, and so forth is started, personalized chronic disease management intervention programs are developed, and the effectiveness of chronic disease management is evaluated. New nurses flow in hospitals. The establishment of hospital chronic disease management and nursing service standards based on PR and the Delphi method that we studied is very different from traditional chronic disease management and nursing. Specific differences are shown in Figure 4.

## 3. Constructing Hospital Chronic Disease Management and Nursing Service Experiments and Conclusions

### 3.1. Degree of Expert Opinion Discussion

In the hospital's chronic disease management and nursing services, the most important thing is the diagnosis and advice from the doctor, which can prescribe the right medicine and carry out the targeted treatment. The degree of discussion of expert opinions is represented by the Kendall coefficient of variation and the coordination coefficient. The coefficient of variation indicates the degree of discussion between experts and indicators. The Kendall tuning factor represents the extent of the doctor's discussion for a certain type of patient. The smaller the coefficient, the higher the degree of coordination among experts, and it is generally believed that the coefficient of variation should be less than 0.25. See Table 1 for details. The degree of authority of an expert determines whether the hospital and the patient's family adopt the doctor's advice. They are relatively convinced in our daily lives. An expert is an authority in an industry, especially in the medical field. After many years of precipitation, the theoretical and practical knowledge is very rich, which is worthy of our trust.

As of 2020, the number of chronic patients in my country increases year by year, as shown in Figure 5. A variety of chronic diseases, including hypertension, hyperlipidemia, fatty liver, diabetes, and so forth, have become the main source of diseases every year in our country. Chronic diseases of both men and women are also the biggest cause of death. Chronic disease is a type of disease that seriously threatens the health of the Chinese people. It has become a major public health problem affecting the country's economic and social development. At present, in terms of prevalence and population, chronic diseases have spread in our country. The main causes of death of patients with chronic diseases in my country are cardiovascular diseases, cancer, and chronic respiratory diseases.

### 3.2. Expert Consultation Index

Expert consultation indicators refer to experts who have not expressed their opinions on the indicators. The average value of the first-level index of expert consultation is 5.47 ~ 5.79 points, the full score rate is 57.37 ~ 88.95%, and the coefficient of variation is 0.19 ~ 0.21. The average value of the second level is that the index significance is 5.26 ~ 5.94 points, the percentage of full marks is 36.32 ~ 94.84%, the coefficient of variation is 0.15 ~ 0.26, the average value of the three levels of index significance is 4.84 ~ 5.89 points, the full score rate is from 20.53% to 89.59%, and the coefficient of variation based on the index selection criteria is 0.16 to 0.28. The two indicators “Awareness rate of chronic disease need management” and “Main approach rate of patients with chronic symptomatic self-monitoring” have a full score of <30%. The team members strictly select indicators and clarify the standard indicators of chronic disease, symptom management, and nursing service items, including 5 first-level indicators, 18 second-level indicators, and 29 third-level indicators. The average distribution of the importance of each index, the full score rate, and the coefficient of variation are shown in Table 2:

With the continuous development of science and technology in our country, the rapid development in all walks of life, especially in the medical field, and the continuous updating of various medical technologies; now, my country's medical field is at the forefront of the world. In terms of self-love, chronic disease management, and nursing, my country has also made great progress in recent years. In many different chronic disease fields, increasingly, experts have emerged, solving a large part of the number of chronic disease patients in my country, as shown in Figure 6. In the past few years, my country has concentrated on the number of chronic disease experts.

In this research, we have invited some Delphi experts, all of whom are very authoritative experts, who are very well known in their fields. Some experts in this survey are very professional in the research of this content and have been engaged in the industry for many years, the theory and practical experience are very rich, they are highly authoritative, and the results of the consultation are relatively reliable.  Table 3 shows the self-evaluation and quantitative results of the familiarity of these experts.

Today, there are more than 400 million chronic disease patients and their families in China. Until 2020, the national mortality rate of chronic diseases is 700 per 100,000 people, that is, 700 deaths out of 100,000 chronic disease patients. The main cause of death in our country is chronic disease.  Figure 7 shows the four types of chronic diseases in the hospital we visited, namely, diabetes, hypertension, stroke, and coronary heart disease. In recent years, the number of chronic disease patients in the hospital has been increasing year by year and has been showing an upward trend.

### 3.3. Hospital Chronic Disease Management and Nursing Service Standards

Based on the above results obtained after expert consultation and expert discussion, the PR team finally discussed and summarized, which was adopted by the hospital. Some chronic disease management and nursing service standards used in the hospital were combined with the hospital's chronic disease management. The current situation, combined with the measurement standards and actual conditions of some other hospitals, has formulated the standards shown in Table 4.

The survey results of Delphi experts found that compared with the results of the first round of research, it can be summarized as follows: the first point of view is more consistent, and only explanatory data are not modified: article 10 is the same as the expert opinion, points 3, 4, and 7, there are also different opinions. Different opinions have professional or regional characteristics. For example, the main content of point 3 is the content of patient evaluation. The two experts with different opinions are both cardiologists, and they think this may be related to the working conditions of the nursing nurses. However, the lack of understanding leading to points 4 and 7 may be due to the nature of the unit. The experts who disagree on these two components are the same, and both come from more specific cardiology hospitals. Therefore, it may lead to inconsistent expert evaluation levels of other general hospitals. Finally, for points 3, 4, and 7, the opinions of most experts were selected. Every expert has different opinions. They contacted the experts again and explained in detail the reasons for their refusal. Experts said they understand and agree. The last round of review was more consistent, but 34 of them still modified the first point. In the second round of the review letter, it was found that all experts agreed with this part of the review and believed that the overall process could be more compact, as shown in Table 5.

## 4. Discussion

In this era, whether for our country or other countries, for our individuals or the society as a whole, chronic disease management and nursing service standards are essential, and they are also an indispensable part of our daily lives. Today, there are more than 400 million chronic disease patients and their families in China. Until 2020, the national mortality rate of chronic diseases was 700 per 100,000 people, that is, 700 deaths out of 100,000 chronic disease patients. The main cause of death in our country is chronic disease. In the past ten years, the prevention and treatment of chronic diseases has attracted wide attention from the medical profession. Various institutions across the country have begun to prevent and treat chronic diseases. The prevention and treatment of chronic diseases is a comprehensive multidisciplinary project, and nursing work is in an advantageous position in the management and nursing of chronic diseases. In the relatively mature chronic disease management model, abroad nursing work runs through the rehabilitation process of all chronic disease patients. However, chronic disease management and nursing services in our country lack a complete and scientific chronic disease management model, and chronic disease treatments are different in different regions, and hospitals also have problems such as inconsistent service content. Also, the main task is not clear; the specific requirements and other issues are not clear. Therefore, to study and establish a unified, standardized, and scientific standard care plan for chronic diseases, objectively guide institutions to provide chronic disease care service plans, comprehensively and scientifically promote the continuous improvement of service items, and help achieve the goal of chronic disease management are an urgent need for our country. In addition, the implementation of a comprehensive management plan for chronic diseases and inter-agency nursing service standards will promote information exchange and promote the arrival of the era of rapid development of chronic diseases.

## 5. Conclusions

This article uses the PR and the Delphi method to conduct a further in-depth study on the current immature chronic disease management and nursing service standards in my country. Managing chronic diseases and subsequent nursing is a difficult task, and due to my country's vast territory, chronic disease management resources and nursing service resources are definitely different in different places. How to meet the needs of patients with chronic diseases while achieving effective management of resources and use, this is what we should think about now. The introduction of chronic disease management and nursing service standards can also promote the development of hospitals as a matter, mission, and important issue. The essence of PR is resource reorganization, and this approach is gradual. The new governance process as an organizational activity is designed to analyze and plan the organizational process in a basic and thorough manner. Related organizational changes are managed to track performance and help the company to grow significantly. Although it is applied to the business model, it is now also applicable to the management of medical and health services. The biggest advantage of the Delphi method is that it is simple and easy to use, without tedious mathematical modeling, and can effectively predict the unknown or future state of the research object in the absence of sufficient statistical data. This research is based on the organizational redesign method, redesigning the new hospital's chronic disease care management process, and consulting experts to determine the chronic disease management plan, indicator system, and related indicators. The plan is used to manage chronic diseases and actual nursing work to achieve further improvements in procedures and plans.

## Figures and Tables

**Figure 1:** PR process entity diagram.

**Figure 2:** Three stages of the PR mode.

**Figure 3:** Schematic diagram of the specific process of the Delphi method.

**Figure 4:** Comparison of the original chronic disease care management process and the new chronic disease care management process.

**Figure 5:** My country's male and female data on chronic diseases.

**Figure 6:** Number of chronic disease experts in my country in recent years.

**Figure 7:** Four trends in the proportion of patients with common chronic diseases in hospitalization.

**Table 1:** Degree of coordination and its significance test results.

Consultation rounds	Project	Coefficient of variation	Coordination coefficient and test results		
			*W* value	Degree of freedom	*P*
First round	First-level indicator	0.09 ~ 0.11	0.204	2	0.021
	Secondary indicators	0.05 ~ 0.16	0.180	12	0.016
	Third-level indicators	0.06 ~ 0.18	0.201	36	0.010
Second round	First-level indicator	0.08 ~ 0.11	0.233	2	0.012
	Secondary indicators	0.05 ~ 0.19	0.250	12	0.019
	Third-level indicators	0.05 ~ 0.16	0.130	35	0.008

**Table 2:** Chronic disease management and nursing service standard program index system.

Index	Importance assignment	Full score ratio (%)	Coefficient of variation
Structure	4.53 + 0.51	52.63	0.11
System construction	4.79 + 0.42	78.95	0.09
Enrollment of patients with chronic diseases	4.58 + 0.51	57.89	0.11
Create personal chronic disease files	4.74 + 0.56	78.95	0.12
Develop a chronic disease management plan and intervene	4.79 + 0.42	78.95	0.09
Evaluation of the effectiveness of chronic disease management	4.84 + 0.37	84.21	0.08

**Table 3:** Expert familiarity self-evaluation and results.

Familiarity	Very familiar	Familiar	General	Unfamiliar	Unfamiliar
Quantitative value	2.0	1.8	1.6	1.4	1.2
Expert frequency	9	8	1	1	1
Points	1.10	1.05	1.0	0.95	0.9
Number of people (*n*)	3	4	3	7	3

**Table 4:** Standard plan of hospital chronic disease management and nursing service.

Field	Dimension	Hospital chronic disease management and nursing service standard plan and its measurement standards
1. Chronic disease management and nursing service organization construction	1.1 Organizational structure	The chief nurse is responsible for the chief supervision, and the chief nurse is responsible for department supervision
	1.2 System construction	The head nurse of each ward is responsible, with 2 nurses assisting
	1.3 Facilities	Complete rate of basic and specialized equipment configuration ≥80%
	1.4 Human Resources	Establishment of admission qualifications for chronic disease nursing staff in various specialties
2. Enrollment of patients with chronic diseases	2.1 Inclusion criteria	All specialties set clear criteria for the inclusion of chronic disease patients
3. Establish personal chronic disease files	3.1 File content	Completion rate of health file content ≥95%
4. Develop a chronic disease management plan and intervene	4.1 Intervention plan	All specialties set up chronic disease intervention plans with specific time points
5. Evaluation of the effectiveness of chronic disease management	5.1 Outcome of the disease	Chronic disease complication rate within 2 years ≤30%

**Table 5:** Investigation results of Delphi experts' supplementary content.

Entry	Main content	Yes		No	
		Frequency	Percentage (%)	Frequency	Percentage (%)
1	Triage time limit	25	95	1	10
2	Process opening	24	94.44	2	7.69
3	Patient assessment content	24	95.55	2	7.86
4	Vital signs measurement	23	89.76	3	14.44
5	Nurse doing electrocardiogram	24	92.22	2	7.52
6	Notice of consultation time	23	87.66	3	18.86
7	Staffing	23	85.69	3	15.96

## Data Availability

The data that support the findings of this study are available from the corresponding author upon reasonable request.
